RETRACTED

# Androgen receptor CAG and GGN repeat length variation contributes more to the tumorigenesis of osteosarcoma

**DOI:** 10.18632/oncotarget.11902

**Published:** 2016-09-08

**Authors:** Yongxiang Shi, Weishan Chen, Qinghuai Li, Zhaoming Ye

**Affiliations:** ^1^ Department of Orthopaedic Surgery, 2nd Affiliated Hospital, School of Medicine, Zhejiang University, Hangzhou, China; ^2^ Department of Medicine, 3rd Hospital of Henan Province, Henan, China

**Keywords:** osteosarcoma, papillary thyroid cancer, AR, repeat, CAG

## Abstract

The androgen receptor (*AR*) is involved in the differentiation and growth of many cancers. We hypothesized that two microsatellite polymorphic variants, *AR* (CAG)n and (GGN)n repeats, were also associated with the development of Papillary thyroid cancer (PTC) and Osteosarcoma. In current study, we conducted two case-control studies in a Chinese population to investigate the possible relationship between these two *AR* repeat polymorphisms and the risk of PTC and Osteosarcoma. The *AR* CAG repeat length was significantly associated with both risk of PTC and Osteosarcoma. Subjects with shorter *AR* CAG repeats had a higher risk of developing PTC (OR = 1.47, 95% CI: 1.17–1.85, *P* = 0.001) and Osteosarcoma (OR = 1.53, 95% CI: 1.19–1.97, *P* = 9.2 × 10^–4^). Specifically, shorter GGN repeats also contribute a significant increased risk of Osteosarcoma (OR = 1.35, 95% CI: 1.03–1.77, *P* = 0.030). Our results contribute to a better understanding of the complex hormone related mechanisms underlying PTC and Osteosarcoma.

## INTRODUCTION

The androgen receptor (*AR*) is involved in the differentiation and growth of many endocrine cancers, including breast cancer, prostate cancer, ovarian cancer, endometrial cancer, bladder cancer, thyroid cancer [1–9]. The *AR* is a nuclear transcription factor that mediates the actions of testosterone and dihydrotestosterone [10]. Two microsatellite polymorphic variants, (CAG)n and (GGN)n repeats, which were located in exon 1 of the *AR* gene, was identified to be associated with the expression level of *AR*, further the development of many endocrine related cancers [10, 11]. Papillary thyroid cancer (PTC) and Osteosarcoma are two kind cancers which have been reported to be associated with sex hormone metabolism [9, 12–14]. Magri et al. [14] identified that AR expressions were associated with a more aggressive phenotype of small T1 differentiated thyroid cancers (DTC). Stanley et al. [9] also found that AR status in thyroid tissues of men and women might predispose to the gender specific incidence of thyroid tumors. DBC1-AR pathways was also identified to be involved in the progression of osteosarcoma [12]. However, to present, no studies have evaluated the associations between the *AR* CAG and GGN repeat length variation and tumorigenesis of PTC and Osteosarcoma.

RETRACTED

Since GGN and CAG repeats could influence the AR protein yield and its transcriptional activity and then paly roles in the tumorigenesis of PTC and Osteosarcoma, thus, in current study, we hypothesized that *AR* (CAG)n and (GGN)n repeats were also associated with the development of PTC and Osteosarcoma. Thus we conducted this case-control study in a Chinese population to first investigate the possible relationships between these two *AR* repeat polymorphisms and the risk of PTC and Osteosarcoma.

## RESULTS

### Characteristics of the studied population

Totally included in the current study were 500 PTC cases and 500 matched healthy controls, as well as 500 Osteosarcoma cases and 500 matched healthy controls (Table 1). Comparing the clinical features between cases and controls, we found a similar age, sex ratio, consumption of tobacco and alcohol in two groups. CAG repeat length ranged from 8 to 33 (median value = 22) among the healthy controls, while GGN repeat length ranged from 15 to 28 (median value = 23) among the healthy controls.

**Table 1:** Comparison of patients and controls by selective characteristics

Variables	PTC			Osteosarcoma		
	Cases (*n* = 500)	Controls (*n* = 500)	*P* value	Cases (*n* = 500)	Controls (*n* = 500)	*P* value
Age (years)	45.7 ± 4.1	45.9 ± 5.2	0.499	28.5 ± 3.5	28.3 ± 3.1	0.339
Gender (female)	375 (75.0%)	359 (71.8%)	0.252	200 (40.0%)	198 (39.6%)	0.897
Smoking status						
Ever	181 (36.2%)	155 (31.0%)	0.082	80 (16.0%)	50 (10.0%)	**0.005**
Never	319 (63.8%)	345 (69.0%)		420 (84.0%)	450 (90.0%)	
Alcohol status						
Ever	331 (66.2%)	329 (65.8%)	0.894	98 (19.6%)	101 (20.2%)	0.812
Never	169 (33.8%)	171 (34.2%)		402 (80.4%)	399 (79.8%)	

### CAG and GGN polymorphisms and PTC risk

We first analyzed the *AR* repeats length as continuous variables. Subjects with shorter AR CAG repeats had a higher risk of developing PTC (OR = 1.16 per 5 repeat decrease, 95% CI: 1.02–1.31, *P* = 0.020). However, shorter *AR* GGN repeats didn't show a significant association with the risk of PTC (*P value* > 0.05). Then, the repeat length was analyzed as categorical variables, and the median value 22, 23 were selected as cut-points for the CAG repeat and the GGN repeat, respectively. As shown in Table 2, compared to those with the longer (≥ 22) CAG repeat length, subjects in the category of shorter (< 22) CAG repeats had a significant 47% increased risk of PTC (OR = 1.47, 95% CI: 1.17–1.85, *P* = 0.001). No significant association was detected for GGN repeat.

**Table 2:** Association of AR repeat length with PTC risk

	Cases, *n* (%)	Controls, *n* (%)	OR (95% CI)*	*P*
**GGN repeat**				
GGN__continous_ (per repeat)			1.04 (0.98–1.11)	0.210
GGN__continous_ (per 5 repeat)			1.22 (0.88–1.69)	0.230
GGN__categorical_				
> 23	160 (32.0%)	174 (34.8%)	Referent	0.320
≤ 23	340 (68.0%)	326 (65.2%)	1.15 (0.87–1.51)	
**CAG repeat**				
GGN__continous_ (per repeat)			1.03 (1.00–1.06)	**0.026**
GGN__continous_ (per 5 repeat)			1.16 (1.02–1.31)	**0.020**
CAG__categorical_				
≥ 22	260 (52.0%)	306 (61.2%)	Referent	**0.001**
< 22	240 (48.0%)	194 (38.8%)	1.47 (1.17–1.85)	

* adjusted by age, gender, smoking status, and alcohol status.

RETRACTED

### CAG and GGN polymorphisms and Osteosarcoma risk

When analyzed as continuous variables, both shorter CAG repeat (OR = 1.40 per 5 repeat decrease, 95% CI: 1.07–1.83, *P* = 0.014) and the GGN repeat (OR = 1.31 per 5 repeat decrease, 95% CI: 1.03–1.67, *P* = 0.029) contribute to higher risk of Osteosarcoma Table 3. Compared to those with the longer (≥ 22) CAG repeat length, subjects in the category of shorter (< 22) CAG repeats had a significant increased risk of Osteosarcoma (OR = 1.53, 95% CI: 1.19–1.97, *P* = 9.2 × 10^–4^). While compared to those with the longer (> 23) GGN repeat length, subjects in the category of shorter (≤ 23) GGN repeats had a significant increased risk of Osteosarcoma (OR = 1.35, 95% CI: 1.03–1.77, *P* = 0.030). Sensitivity analyses were also conducted to eliminate the subjects with extreme age, however, the significant associations were not affected.

**Table 3:** Association of AR repeat length with Osteosarcoma risk

	Cases, *n* (%)	Controls, *n* (%)	OR (95% CI)*	*P*
**GGN repeat**				
GGN__continous_ (per repeat)			1.09 (1.01–1.18)	**0.032**
GGN__continous_ (per 5 repeat)			1.31 (1.03–1.67)	**0.029**
GGN__categorical_				
> 23	148 (29.6%)	180 (36.0%)	Referent	**0.030**
≤ 23	352 (70.4%)	320 (64.0%)	1.35 (1.03–1.77)	
**CAG repeat**				
GGN__continous_ (per repeat)			1.07 (1.01–1.13)	**0.019**
GGN__continous_ (per 5 repeat)			1.40 (1.07–1.83)	**0.014**
CAG__categorical_				
≥ 22	248 (48.4%)	294 (58.8%)	Referent	**9.2 × 10^−4^**
< 22	258 (51.6%)	206 (41.2%)	1.53 (1.19–1.97)	

* adjusted by age, gender, smoking status, and alcohol status.

## DISCUSSION

To the best of our knowledge, this is the first report to attempt an evaluation of the associations of *AR* repeats length potentially related to PTC and Osteosarcoma carcinogenesis. We identified that subjects with shorter *AR* repeats length contributed to higher risk of developing PTC and Osteosarcoma, either as continuous variable or a categorical variable, which indicating the robustness of the results in current study.

*AR* may act by a no-genomic pathway that entails the rapid activation of kinase-signaling cascades and the modulation of intracellular calcium levels [15]. Previous studies have found *AR* repeats length could influence development, migration and invasion of metastasis of many endocrine related cancers [16, 17]. Zhang et al. [18] also identified that *AR* promotes gastric cancer cell migration and invasion via AKT-phosphorylation dependent up-regulation of matrix metalloproteinase 9, and its expression was positively correlated with lymph node metastasis and late TNM stages. The CAG repeat length of *AR* inversely affects its transactivation potential, either as a directly altered receptor function or indirectly reduced *AR* messenger in RNA and protein levels [19]. Early in 1996, Rossi et al has confirmed the androgen receptor gene expression in human thyroid cells and tumors [20]. The thyroid hormone could also affect androgen receptor messenger RNA expression [21]. Sex steroid receptors including estrogen receptors (ER), progesterone receptors (PR), and AR have been sporadically reported in human osteosarcoma or its cell lines [22]. DBC1/CCAR2 was identified to be involved in the stabilization of androgen receptor and the progression of osteosarcoma [12]. All evidence above revealed potential essential role of *AR* among the tumorigenesis of PTC and Osteosarcoma.

RETRACTED

In current study, we found that subjects with shorter *AR* CAG repeats had a higher risk of developing PTC (OR = 1.47, 95% CI: 1.17–1.85, *P* = 0.001) and Osteosarcoma (OR = 1.53, 95% CI: 1.19–1.97, *P* = 9.2 × 10^–4^). While compared to those with the longer (> 23) GGN repeat length, subjects in the category of shorter (≤ 23) GGN repeats had a significant increased risk of Osteosarcoma (OR = 1.35, 95% CI: 1.03–1.77, *P* = 0.030). These findings were consistent with previous studies about epithelial ovarian cancer [23, 24], TMPRSS2:ERG-positive prostate cancer [25], breast cancer [26, 27], prostate cancer [28], and so on. Major strength of the current study was the large sample size to minimize type I error. Some limitations should also be addressed when interpret the results in current study. First, we could not rule out the influence of selection bias because of the natural of retrospective study design. However, we have selected the controls which were frequency-matched with cases by age at cancer diagnosis and gender, which aims to reduce the bias. Second, we didn't evaluated the gene-environment interaction for PTC and Osteosarcoma risk.

In summary, our study supported short *AR* CAG repeat length as a susceptible factor for PTC and Osteosarcoma risk in Chinese population. Our results contribute to a better understanding of the complex hormone related mechanisms underlying tumorigenesis and add to the current state of knowledge regarding the susceptibility of *AR* to PTC and Osteosarcoma. However, further prospective studies with larger sample size involving different ethnicities, as well as further functional studies, are needed to confirm our findings.

RETRACTED

## MATERIALS AND METHODS

### Subjects

In current study, the patients were recruited from May, 2010, and diagnosed by surgical operation. Controls were recruited from the general population living in the same areas and matched with cases by age at cancer diagnosis and gender. The medical records of healthy controls were also reviewed to ensure that they have no previous or current diagnosis of cancers or related diseases. All participants were interviewed face-to-face by trained professionals (nurses or medical staff) using a structured questionnaire. After the interview, 5 milliliters of peripheral blood was collected from each subject in our study. Both approval from the appropriate institutional review board and written informed consents from patients who were included in this study were obtained.

### Microsatellite analysis of *AR* repeat length and quality control

Genomic DNA was extracted from peripheral blood samples using the Qiagen Blood Kit (Qiagen, Chatsworth, CA, USA) according the instructions of manufacturer. The two *AR* repeat region was amplified by PCR from 50 ng template DNA using primers flanking the *AR* repeat in exon 1 (For CAG repeat: F: 5′-ACCCA GAGGCCGCGAGCGCAG- 3′ and R: 5′-TTGCTGTTCCT CATCCAGGA-3′; for GGN repeat: F: 5′-CGGTTCTGG GTCACCCTC A-3′ and R: 5′-TCACCATGCCGCCAG GGTA-3′). Then the fragments were tested on denaturing polyacrylamide gels, and PCR products were purified and sequenced using the Applied Biosystems Prism 3700XL and analyzed by Applied Biosystems Prism Genescan automated fluorescence detection (Applied Biosystems, Foster City, CA). Positive and negative control was used for quality control, and the concordance rate was 100%.

### Statistical analyses

Difference of clinical characteristics (age, sex, smoking and alcohol status) between PTC cases and controls were tested by chi-square test or *t-test*. For the *AR* repeat lengths comparison, the Shapiro-Wilk test was used to verify the normality of distribution, and Levene's test for equality of variances. When the assumptions were met, *t-test* was used to test the differences for the *AR* repeat lengths. Or, the Mann-Whitney *U* test was used. Unconditional logistic regression was used to calculate odds ratios (ORs) as well as confidence intervals (CIs) for PTC risk associated with repeat genotypes. We identified the cut-points (median value) on the basis of repeat number distribution in the control group. All statistical analyses were performed using SAS 9.2 (SAS Institute, Cary, NC, USA). Statistical significance was determined according to the conventional significance-level of α = 5%.
